# 6′-O-Galloylpaeoniflorin Exerts Inhibitory Bioactivities in Human Neuroblastoma Cells via Modulating AMPK/miR-489/XIAP Pathway

**DOI:** 10.1155/2022/1327835

**Published:** 2022-05-05

**Authors:** Lijun Zhou, Aiwu Li, Qiangye Zhang

**Affiliations:** Department of Pediatric Surgery, Qilu Hospital of Shandong University, Jinan 250012, China

## Abstract

Although therapies against neuroblastoma (NBM) have advanced, the patients still suffer from poor prognoses due to distal metastasis or the occurrence of multidrug resistance. Accumulating evidence has proved that chemicals derived from natural products possess potent anti-NBM properties or can be used as adjuvants for chemotherapy. In the present study, we demonstrated that 6′-O-galloylpaeoniflorin (GPF), a galloylated derivative of paeoniflorin isolated from the roots of *Paeonia lactiflora Pall*, exerted significant inhibitory effects on proliferation and invasion of SH-SY5Y cells (an NBM cell line) and enhanced the sensitivity of SH-SY5Y cells to cisplatin in vitro. Further studies showed that GPF treatment upregulated miR-489 in NBM cells via activating AMP-activated protein kinase (AMPK). We also demonstrated that similar to GPF treatment, miR-489 exhibited a significant anti-NBM capacity. Further studies showed that miR-489 directly targeted the X-linked inhibitor of apoptosis protein (XIAP). Overall, our results indicated that GPF possessed an evident anti-NBM capacity dependent on AMPK/miR-489/XIAP pathway, providing an emerging strategy for clinical treatment of NBM.

## 1. Introduction

As one of the most frequent malignancies in infants and young children, neuroblastoma (NBM) accounts for about 15% of cancer-related mortality in the pediatric population [1]. Therapeutic approaches for NBM include surgery, chemotherapy, radiotherapy, and/or stem cell transplantation [2]. Unfortunately, although modest improvements have yielded in the prognosis of NBM patients with common treatments, the median overall survival (OS) in drug-resistant NBM remains poor [3]. Recently, more and more attention has been paid to the precise molecular regulatory mechanisms in the tumorigenesis of NBM, aiming at developing novel effective diagnostic and therapeutic strategies [4–6].

Since ancient times, natural compounds have been applied to cure disorders [7]. Accumulating evidence has proved the efficiency of natural compound-based strategies in the treatment of human diseases, such as asthma [8, 9], infection [10], diabetes mellitus, neurological disease [11, 12], and various types of tumors [13, 14]. These compounds present as chemotherapeutic agents independently and can be used as adjuvants for chemotherapy or radiotherapy [13]. For example, isatin has been reported to arrest the proliferation and promote apoptosis in NBM cell line SH-SY5Y cells [15]. Gallic acid, epigallocatechin-3-gallate, and curcumin enhance cisplatin-induced apoptosis in non-small-cell lung cancer (NSCLC) cells via activating proapoptotic signaling and antagonism of the antiapoptotic proteins [16–18]. Oleanolic acid, as well as ursolic acid and micheliolide, enhance the radiosensitivity of NSCLC cells via accelerating the degradation of HIF-1*α* [19–21]. Therefore, natural compounds are expected to become potential anti-NBM chemicals [22].

As a family of endogenous short RNAs (18-25 nt), microRNAs (miRNAs) regulate the expressions of their cellular targets through binding to the 3′-untranslated region (3′-UTR) of mRNA [23, 24]. Studies have identified that miRNAs are implicated in regulating over 60% of human coding genes [25]. miRNAs function extensively in a wide range of cellular biological and pathophysiological processes, such as embryonic development [26], differentiation [27], inflammation [28], and carcinogenesis [29]. In addition, accumulating evidence has emphasized the critical role of miRNAs in various malignant neoplasms, including NBM [6]. Intriguingly, some natural compounds have been demonstrated to exert their pharmacological effects by regulating the expressions of miRNAs [30]. For instance, osthole inhibits the expression of miRNA-22-3p in pulmonary artery smooth muscle cells, restoring the dysregulated lipid metabolism, which alleviates pulmonary vascular remodeling in pulmonary arterial hypertension [31]. 6′-O-Galloylpaeoniflorin (GPF) is a galloylated derivative of paeoniflorin isolated from the roots of *Paeonia lactiflora Pall*, which possesses therapeutic effects in treating cerebral infarct [11], osteoporosis [32], and lung cancer [33]. GPF can upregulate miR-299-5p via activating the AMP-activated protein kinase (AMPK) pathway and downregulate ATF2, resulting in the suppressed proliferation and invasion in NSCLC cell lines, A549, and H1299 cells [33]. However, whether GPF possesses an anti-NBM capacity remains largely unexplored.

Based on the abovementioned evidence, we aimed to clarify the role of GPF in treating NBM in the present study. Our findings showed that GPF treatment remarkably restrained the proliferation and invasion of NBM cell line SH-SY5Y cells and enhanced the chemosensitivities of SH-SY5Y cells to cisplatin. The results also demonstrated that the expression of a tumor-suppressive miRNA, miR-489, was increased in response to treatment of GPF, which was primed by AMPK activation. Further studies identified that the agonism of miR-489 could reduce proliferation and enhance cisplatin-induced apoptosis in NBM cells. Additionally, we revealed that the X-linked inhibitor of apoptosis protein (XIAP), a critical oncogene, was a cellular target of miR-489 in SH-SY5Y cells. Collectively, our findings provided valuable insights into the pharmacological effects of GPF, highlighting its therapeutic potential in the treatment of NBM by regulating the expression of XIAP.

## 2. Materials and Methods

### 2.1. Cell Culture

The human NBM cell line SH-SY5Y was kindly gifted by Dr. Hao at Jilin University. Cells were maintained in Dulbecco's Modified Eagle Medium (DMEM, Gibco) supplemented with 10% fetal bovine serum (FBS, Sigma) at 37°C in a humidified atmosphere containing 5% CO_2_.

### 2.2. miRNA Transfection

The miR-489 and negative control were purchased from RiboBio Co. (Guangzhou, China) and transfected into SH-SY5Y cells as previously described [34]. Briefly, digested cells were prepared as a single-cell suspension and then plated at appropriate densities. When a confluence of 80% was achieved, miR-489 or the negative miRNA was added to each well at a final concentration of 50 nM.

### 2.3. Cell Proliferation Test

Cell Counting Kit-8 (CCK-8; Sigma-Aldrich) assay was performed to assess the proliferation rate of SH-SY5Y cells in vitro. Briefly, after transfection with miR-489 or scramble control, cells (3 × 10^3^ cells/mL) were seeded into 96-well plates. After 24, 48, and 72 h of incubation, 10 *μ*L CCK-8 solution was added to each well, followed by incubation for another 90 min. The OD at a wavelength of 450 nm was determined using a BioTek Synergy H1 microplate reader.

### 2.4. Colony Formation Assay

The colony formation assay was performed to evaluate the cell survival in vitro as previously described [34]. Briefly, SH-SY5Y cells were seeded into 6-well plates (300 cells/well) and cultured at 37°C in a humidified atmosphere containing 5% CO_2_ for 10 days. Subsequently, the culture medium was discarded, and 0.1% crystal violet (Beyotime, Haimen, China) was used to stain the cells. Colonies of greater than 64 cells were counted.

### 2.5. Cell Apoptosis Assay

Cell apoptosis was assessed using an Annexin V/propidium iodide (PI) kit (Beyotime, Haimen, China) according to the manufacturer's instructions. After miR-489 or the scramble miRNA transfection, SH-SY5Y cells were digested using 0.25% Trypsin (Invitrogen) and washed three times. Subsequently, the cells were resuspended in provided staining buffer, followed by incubation with Annexin V for about 1 h. Then, the cells were incubated with PI for another 5 min. The proportion of apoptotic cells was determined by flow cytometry (Beckman CytoFLEX).

### 2.6. Cell Scratch Assay

Cell scratch assay was conducted to determine the migratory ability of SH-SY5Y cells as previously described [35]. Briefly, cells were prepared as a single-cell suspension and then seeded into 6-well plates. When a confluence of approximately 80% was achieved, the cell monolayer was scratched to create a “wound.” Next, the cells were cultured with a culture medium supplemented with 1% FBS at 37°C in a humidified atmosphere containing 5% CO_2_ for 2 and 24 h. Subsequently, the width of the wound was examined using an inverted microscope (Olympus).

### 2.7. Transwell Assay

A transwell assay was conducted to evaluate the migratory capacity of SH-SY5Y cells as previously reported [36]. Briefly, cells were seeded into a Millicell cell culture insert (Millipore) containing 100 *μ*L serum-free medium at a density of 10^5^ cells/mL. Then, the insert was added to a 24-well plate containing 100 *μ*L DMEM (10% FBS) in each well. Then, the plate was incubated at 37°C. After 1 day, the medium was discarded, and the membrane of the chamber was removed, followed by staining using 0.5% crystal violet solution. The migrated cells were photographed using an Olympus MX40 inverted microscope and quantified by counting six randomly selected fields. To assess the cell invasive ability, the bottom of the cell culture insert was coated with Matrigel (Corning) prior to the migration assay.

### 2.8. Quantitative PCR (qPCR)

Total RNA was extracted from SH-SY5Y cells using Biomarker total RNA isolation kit. Purified RNA was reversely transcribed to cDNA with MonScript™ RTIII Super Mix with dsDNase (Monald, Wuhan, China) according to the manufacturer's instructions. qPCR assay was performed to determine the expressions of mRNAs and miRNAs using MonAmp™ Fast SYBR® Green qPCR Mix (Monald) on a Bio-Rad CFX Connect PCR System. The primers of XIAP and housekeeping gene GAPDH were listed as follows:

XIAP-forward: 5′-AAGAGAAGATGACTTTTAACAG-3′, XIAP-reverse: 5′-TGCTGAGTCTCCATATTGCC-3′; GAPDH-forward: 5′-GCGAGATCGCACTCATCATCT-3′, GAPDH-reverse: 5′-TCAGTGGTGGACCTGACC-3′.

The relative expressions of the target mRNA and miRNA were calculated using the 2^-*ΔΔ*Ct^ method [37].

### 2.9. Immunoblotting Analysis

Total protein was isolated from SH-SY5Y cells using Tris-NaCl buffer (50 mM Tris, 150 mM NaCl) containing 1% Triton. The expression of XIAP at the protein level was semiquantitated by the Western blotting analysis as previously described [38]. Briefly, equal amounts of proteins were subjected to sodium dodecyl sulfate-polyacrylamide gel electrophoresis (SDS-PAGE) on 10% gels and then electrotransferred onto the polyvinylidene difluoride membranes. The blots were blocked in PBS containing Tween-20 (PBST) supplemented with 1% bovine serum albumin, followed by incubation with primary antibodies against *α*-XIAP (Abcam, ab229050, 1 : 3,000) and *α*-GAPDH (Abcam, ab8245, 1 : 5,000) overnight at 4°C. Subsequently, the blots were washed with PBST and incubated with horseradish peroxidase-labeled secondary antibodies (1 : 5,000) at room temperature for 2 h. The immunoreactive bands were visualized using the Bio-Rad ChemiDoc Touch System.

### 2.10. Luciferase Assay

Luciferase assay was conducted to validate the interaction between miR-489 and 3′UTR of XIAP as previously reported [39]. Briefly, the 3′UTR of XIAP was cloned into the pmirGLO vector, termed XIAP 3′UTR-wt. Mutation in the predicted miR-489 binding site was introduced using the Quikchange kit (Agilent, cat.# 600670), which was set as a negative control (XIAP 3′UTR-mut). Either miR-489 or the scramble control was cotransfected with the reporter plasmids (Invitrogen) into SH-SY5Y cells. After 48 h of transfection, the cell luciferase activity was determined using a BioTek Synergy H1 microplate reader.

### 2.11. Statistical Analysis

Statistical analysis was performed using GraphPad Prism 8.0. A *p* < 0.05 was considered statistically different.

## 3. Results

### 3.1. GPF Treatment Inhibits Proliferation and Restores Chemosensitivity in SH-SY5Y Cells

The pharmacological effects of GPF on the proliferation of NBM were determined using a CCK-8 assay. The results indicated that GPF treatment dose-dependently decreased the proliferation of SH-SY5Y cells in vitro (Figure 1(a)). Consistently, the colony formation assay showed that GPF treatment dose-dependently inhibited the colony formation of SH-SY5Y cells (Figure 1(b)). To determine the effects of GPF on chemosensitivity in NBM, SH-SY5Y cells stimulated with or without GPF were subjected to cisplatin treatment, and then the proportion of apoptotic SH-SY5Y cells was determined by Annexin V-FITC/PI staining. Fewer apoptotic cells were detected in untreated or GPF-treated cells, whereas about 17% of apoptotic cells were detected in the cisplatin treatment (Figure 1(c)). Intriguingly, as shown in Figure 1(c), pretreatment with GPF significantly enhanced the cisplatin-induced apoptosis. These results indicated that GPF exerted antiproliferation and proapoptotic capacity in NBM cells.

### 3.2. Treatment with GPF Restrains the Migratory and Invasive Ability of SH-SY5Y Cells

The pharmacological effects of GPF treatment on the migratory and invasive ability of NBM cells were evaluated by cell scratch and transwell assays in SH-SY5Y cells.  Figure 2(a) shows that the wound healing rate of SH-SY5Y cells treated with GPF was significantly lower compared with untreated cells (Figure 2(a)). In addition, the transwell assay demonstrated that GPF treatment significantly reduced the migratory and invasive capacity of SH-SY5Y cells (Figures 2(b) and 2(c)) in a dose-dependent manner. These results indicated that GPF possessed suppressive effects on the migratory and invasive ability of NBM cells in vitro.

### 3.3. GPF Treatment Upregulates the Expressions of miR-489 Dependent on AMPK Activation

A previous study has demonstrated that GPF treatment induces AMPK activation in NSCLC A549 and H460 cells. Consistently, we found that GPF treatment also activated AMPK in SH-SY5Y cells in a dose-dependent manner, which could be retarded by AMPK antagonist compound C (Figure 3(a)). Intriguingly, we also found that treatment with GPF remarkably enhanced the expression of a tumor suppressor, miR-489, in SH-SY5Y cells in a dose- and time-dependent manner (Figure 3(b)). Besides, the upregulation of miR-489 induced by GPF treatment was markedly blocked by compound C (Figure 3(c)). These results suggested that GPF induced an AMPK-dependent upregulation of miR-489 in NBM cells.

### 3.4. miR-489 Induces Proliferation Arrest and Apoptosis in NBM Cells

The role of miR-489 in the proliferation of NBM cells was determined using a CCK-8 assay. The results indicated that the proliferation of SH-SY5Y cells transfected with miR-489 was decreased compared with those transfected with scramble miRNAs (Figure 4(a)). Furthermore, the colony formation assay suggested that enforced expression of miR-489 decreased the number of cell colonies compared with the scramble miRNA (Figure 4(b)). Additionally, the apoptosis assay demonstrated that SH-SY5Y cells transfected with miR-489 displayed higher apoptotic rates compared with those transfected with the scramble miRNA in response to cisplatin treatment (Figure 4(c)). These findings manifested that miR-489 played a regulatory role in the proliferation, survival, and apoptosis of NBM cells.

### 3.5. miR-489 Restrains the Migratory and Invasive Ability of SH-SY5Y Cells

The role of miR-489 in the migratory and invasive ability of NBM cells was evaluated by cell scratch and transwell assays in SH-SY5Y cells. The enhanced expression of miR-489 remarkably reduced the wound healing rate compared with scramble miRNA-treated cells (Figure 5(a)). Additionally, the transwell assay demonstrated that miR-489 transfection reduced the migratory (Figure 5(b)) and invasive (Figure 5(c)) capacity of SH-SY5Y cells. These findings indicated that miR-489 functioned as a suppressor in regulating migration and invasion of NBM cells in vitro.

### 3.6. miR-489 Targets XIAP and Decreases Its Expression in NBM Cells

Bioinformatic analysis using two predictive algorithms, TargetScan and http://microRNA.org, was performed to further explore the genes targeted by miR-489 in NBM cells. The results revealed a potential miR-489 binding site within the 3'UTR of XIAP, a potent antiapoptotic adaptor (Figure 6(a)). The luciferase assay indicated that miR-489 transfection inhibited the activities of luciferase in SH-SY5Y cells transfected with plasmids expressing 3′UTR of XIAP, but not the 3′UTR mutants (Figure 6(b)). Furthermore, the overexpression of miR-489 downregulated the expression of XIAP at the mRNA level in SH-SY5Y cells (Figure 6(c)). Consistently, miR-489 transfection downregulated the expression of XIAP at the protein level in NBM cells (Figure 6(d)). Taken together, these findings suggested that miR-489 bound to 3′UTR of XIAP mRNA for degradation, thus regulating its expression.

## 4. Discussion

Up to date, the most well-documented pharmacological effect of GPF is its antioxidant capacities. In vitro, GPF exerts a practical radical scavenging effect due to its multiple phenolic hydroxyl groups [40] and rescues human keratinocyte cell line HaCaT cells from ultraviolet-induced apoptosis via scavenging reactive oxygen species (ROS) [41]. Besides the intrinsic capacity to eliminate free radicals, GPF treatment significantly attenuates oxidative stress induced by cerebral ischemia-reperfusion through the nuclear factor erythroid 2-related factor 2 (NRF2) pathway [11]. However, the pharmacological effects of GPF on cancer remain largely unexplored. In the present study, we aimed to reveal a novel function of GPF. We found that treatment with GPF remarkably arrested the proliferation, suppressed the invasion, and enhanced chemosensitivity in NBM cells at a dosage that was not toxic to normal cells.

A previous study has reported that GPF treatment upregulates the expression of miR-299-5p to downregulate activating transcription factor 2 (ATF2), thus leading to inhibited progression of NSCLC cells [33]. Intriguingly, we demonstrated that upregulation of miR-489 induced by GPF was implicated in its anti-NBM capacity. Furthermore, it has been reported that GPF remarkably induces the phosphorylation of AMPK, resulting in Nrf2/HO-1 pathway activation [11]. We also observed that GPF treatment induced phosphorylation of AMPK in NBM cells. Intriguingly, pretreatment with compound C, an AMPK antagonist, significantly reduced the upregulation of miR-489 induced by GPF, indicating that this effect of GPF was AMPK dependent.

Accumulating evidence indicates that dysregulation of miR-489 is a common event in tumorigenesis, and it functions as a potent suppressor in growth and metastasis in various malignancies, including breast cancer [42], glioma [43], hepatoma [44], and bladder cancer [45]. In addition, Chen et al. have reported that miR-489 modulates chemosensitivity in human breast cancer cells [46], and upregulation of miR-489 restores the cisplatin chemosensitivity in ovarian cancer cells via directly targeting Akt3 for degradation [47]. To date, very few studies have explored the role of miR-489 in NBM. As complementary information, we provided dramatic biological evidence that miR-489 could arrest the proliferation and promote apoptosis of NBM cells, indicating the antioncogenic property of miR-489 in the NBM.

It has been reported that miR-489 can promote apoptosis in glioma cells via inhibiting the SPIN1-priming PI3K/AKT pathway [43]. Similarly, our findings revealed that the overexpression of miR-489 could also induce compelling apoptosis in NBM cells in vitro. To further explore the mechanism underlying the antiapoptotic effects of miR-489, we first identified XIAP as a bona fide target of miR-489. XIAP, also known as an inhibitor of apoptosis protein 3 (IAP3), is one of the most potent members of the human inhibitor of apoptosis protein (IAP) family, which consists of eight members [48]. Dysregulation of XIAP has been found in several malignancies, including thyroid carcinoma [49], lymphoma [50], and glioma [51]. Furthermore, XIAP hyperexpression accelerates the tumor growth and induces blockage of apoptosis, leading to the development and progression of cancer [52]. XIAP exerts its antiapoptotic function through inhibiting caspases 3, 7, and 9 [53, 54], accounting for the proapoptotic effects of miR-489 indicated in our study.

There are still limitations in this study. First, the precise mechanism underlying the GPF-induced expression of miR-489 is still elusive, though our results indicated that the AMPK pathway was involved in this process. AMPK can interact with diverse signaling pathways, such as the Nrf2 pathway, autophagy, PI3K/Akt pathway, and the mitogen-activated protein kinase (MAPK) pathway. The direct downstream pathway of AMPK mediating miR-489 upregulation needs to be further elucidated. Finally, although miR-489 exerted anti-NBM effects, its contributions to the tumor-suppressive capabilities of GPF are not well documented. Therefore, additional experiments, such as the usage of miR-489 inhibitors, should be carried out to determine the role of miR-489 in the anti-NBM properties of GPF.

In conclusion, our findings presented that GPF was a novel AMPK agonist, which regulated miR-489/XIAP. Through this mechanism, GPF exhibited significant capacity in suppressing the progression of NBM in vitro (Figure 7). These results indicated that GPF could be used as an alternative to the current treatment of NBM and highlighted the potential value of targeting the AMPK/miR-489/XIAP axis in the development of new approaches against NBM.

## Figures and Tables

**Figure 1:** GPF treatment inhibits the proliferation and survival of NBM cells. SH-SY5Y cells were treated with indicated doses of GPF. (a) At 24 h posttreatment, the CCK-8 assay was conducted to evaluate the proliferation of SH-SY5Y cells. (b) At 10 days post-GPF treatment, SH-SY5Y cells were stained with crystal violet, and the number of cell colonies was calculated. (c) At 24 h after treatment, SH-SY5Y cells were treated with cisplatin (5 *μ*M) or the vehicle for another 24 h, followed by apoptosis assay. *p* values: ^∗^*p* < 0.05; ^∗∗^*p* < 0.01 (versus the control group without any treatment).

**Figure 2:** GPF treatment inhibits the migratory and invasive ability of NBM cells. SH-SY5Y cells were treated with the indicated concentrations of GPF for 24 h. (a) The migratory ability of SH-SY5Y cells was evaluated by a cell scratch test. The migratory and invasive abilities of SH-SY5Y cells were evaluated by transwell migration (b) and invasion (c) assays. ^∗^*p* < 0.05; ^∗∗^*p* < 0.01.

**Figure 3:** GPF treatment increases the expression of miR-489 in NBM cells. (a) SH-SY5Y cells were treated with the indicated concentrations of GPF. At 6 h after GFP treatment, phosphorylated AMPK in cells was detected by immunoblotting. (b) SH-SY5Y cells were treated with the indicated concentrations of GPF for 24 h or 100 *μ*M GPF for different durations. The expression of miR-489 was determined by qPCR. (c) After pretreatment with or without compound C for 6 h, SH-SY5Y cells were exposed to GPF treatment for another 18 h, and the expression of miR-489 was determined by qPCR. ^∗^*p* < 0.05; ^∗∗^*p* < 0.01.

**Figure 4:** Transfection with miR-489 inhibits the proliferation and survival of NBM cells. Either miR-489 or scramble miRNA was transfected into SH-SY5Y cells. (a) At 24 h, 48 h, and 72 h post-miR-489 transfection, the CCK-8 assay was conducted to evaluate SH-SY5Y proliferation. (b) At 10 days post-GPF treatment, SH-SY5Y cells were stained with crystal violet, and the number of cell colonies was calculated. (c) At 48 h after transfection, SH-SY5Y cells were treated with cisplatin (5 *μ*M) or the vehicle for another 24 h, followed by an apoptosis assay. ^∗^*p* < 0.05, ^∗∗^*p* < 0.01.

**Figure 5:** miR-489 inhibits the migratory and invasive ability of NBM cells. Either miR-489 or scramble miRNA was transfected into SH-SY5Y cells. (a) The migratory ability of SH-SY5Y cells was evaluated by a cell scratch test. The migratory and invasive abilities of SH-SY5Y cells were evaluated by transwell migration (b) and invasion (c) assays. ^∗^*p* < 0.05; ^∗∗^*p* < 0.01.

**Figure 6:** miR-489 targets XIAP 3′UTR. (a) The binding site of miR-489 and its mutants within the XIAP mRNA 3′UTR were shown. (b) miR-489 or scramble miRNA was cotransfected into NBM cells with pMIR-REPORT (vector), recombinant pMIR-REPORT expressing 3 ′ UTR-wt, or the mutants, respectively. The luciferase activity in cells was determined at 48 h after transfection. Either miR-489 or scramble miRNA was transfected into SH-SY5Y cells. The expression of XIAP at the mRNA (c) and protein (d) levels was determined at 48 h after transfection by qPCR and immunoblotting, respectively. ^∗^*p* < 0.05; ^∗∗^*p* < 0.01.

**Figure 7:** Schematic diagram depicting the anti-NBM effects of GPF.

## Data Availability

All data used to support the findings of this study are included within the article.

## References

[1] Colon N. C., Chung D. H. (2011). Neuroblastoma. *Adv Pediatr*.

[2] Bhoopathi P., Mannangatti P., Emdad L., Das S. K., Fisher P. B. (2021). The quest to develop an effective therapy for neuroblastoma. *Journal of Cellular Physiology*.

[3] Abdelmeguid A. S., Bell D., Roberts D. (2022). Long-term outcomes of olfactory neuroblastoma: MD Anderson Cancer Center Experience and Review of the Literature. *Laryngoscope*.

[4] Huang S., Gong N., Li J. (2022). The role of ncRNAs in neuroblastoma: mechanisms, biomarkers and therapeutic targets. *Biomarker Research*.

[5] Stainczyk S. A., Westermann F. (2022). Neuroblastoma—Telomere maintenance, deregulated signaling transduction and beyond. *International Journal of Cancer*.

[6] Veeraraghavan V. P., Jayaraman S., Rengasamy G., Mony U., Ganapathy D. M. (2022). Deciphering the role of microRNAs in neuroblastoma. *Molecules*.

[7] Chopra B., Dhingra A. K. (2021). Natural products: a lead for drug discovery and development. *Phytotherapy Research*.

[8] Zhu Y., Sun D., Liu H. (2021). Bixin protects mice against bronchial asthma though modulating PI3K/Akt pathway. *International Immunopharmacology*.

[9] Zhu Y., Wang C., Luo J. (2021). The protective role of Zingerone in a murine asthma model via activation of the AMPK/Nrf2/HO-1 pathway. *Food & Function*.

[10] Zhang Y., Liu Y., Luo J., Jie J., Deng X., Song L. (2021). The herbal compound thymol targets multiple salmonella typhimurium virulence factors for Lon protease degradation. *Frontiers in Pharmacology*.

[11] Wen Z., Hou W., Wu W. (2018). 6'-O-Galloylpaeoniflorin attenuates cerebral ischemia reperfusion-induced Neuroinflammation and oxidative stress via PI3K/Akt/Nrf2 activation. *Oxidative Medicine and Cellular Longevity*.

[12] Song L., Li X., Bai X. X., Gao J., Wang C. Y. (2017). Calycosin improves cognitive function in a transgenic mouse model of Alzheimer's disease by activating the protein kinase C pathway. *Neural Regeneration Research*.

[13] Wen T., Song L., Hua S. (2021). Perspectives and controversies regarding the use of natural products for the treatment of lung cancer. *Cancer Medicine*.

[14] Lichota A., Gwozdzinski K. (2018). Anticancer activity of natural compounds from plant and marine environment. *International Journal of Molecular Sciences*.

[15] Xu P., Hou L., Ju C. (2016). Isatin inhibits the proliferation and invasion of SH-SY5Y neuroblastoma cells. *Molecular Medicine Reports*.

[16] Chanvorachote P., Pongrakhananon V., Wannachaiyasit S., Luanpitpong S., Rojanasakul Y., Nimmannit U. (2009). Curcumin sensitizes lung cancer cells to cisplatin-induced apoptosis through superoxide anion-mediated Bcl-2 degradation. *Cancer Investigation*.

[17] Wang R., Ma L., Weng D., Yao J., Liu X., Jin F. (2016). Gallic acid induces apoptosis and enhances the anticancer effects of cisplatin in human small cell lung cancer H446 cell line via the ROS-dependent mitochondrial apoptotic pathway. *Oncology Reports*.

[18] Zhang Y., Wang X., Han L., Zhou Y., Sun S. (2015). Green tea polyphenol EGCG reverse cisplatin resistance of A549/DDP cell line through candidate genes demethylation. *Biomedicine & Pharmacotherapy*.

[19] Qi R., Jin W., Wang J. (2014). Oleanolic acid enhances the radiosensitivity of tumor cells under mimetic hypoxia through the reduction in intracellular GSH content and HIF-1*α* expression. *Oncology Reports*.

[20] Song B., Zhang Q., Yu M. (2017). Ursolic acid sensitizes radioresistant NSCLC cells expressing HIF-1*α* through reducing endogenous GSH and inhibiting HIF-1*α*. *Oncology Letters*.

[21] Kong P., Yu K. N., Yang M. (2020). Micheliolide enhances radiosensitivities of p53-deficient non-small-cell lung cancer via promoting HIF-1*α* degradation. *International Journal of Molecular Sciences*.

[22] Patiño-Morales C. C., Jaime-Cruz R., Sánchez-Gómez C. (2022). Antitumor effects of natural compounds derived from Allium sativum on neuroblastoma: an overview. *Antioxidants (Basel)*.

[23] Seok H., Ham J., Jang E. S., Chi S. W. (2016). MicroRNA target recognition: insights from transcriptome-wide non-canonical interactions. *Molecules and Cells*.

[24] Chaudhuri K., Chatterjee R. (2007). MicroRNA detection and target prediction: integration of computational and experimental approaches. *DNA and Cell Biology*.

[25] Leclercq M., Diallo A. B., Blanchette M. (2017). Prediction of human miRNA target genes using computationally reconstructed ancestral mammalian sequences. *Nucleic Acids Research*.

[26] Kasper D. M., Moro A., Ristori E. (2017). MicroRNAs establish uniform traits during the architecture of vertebrate embryos. *Developmental Cell*.

[27] Gu Y., Ma L., Song L., Li X., Chen D., Bai X. (2017). miR-155 inhibits mouse osteoblast differentiation by suppressing SMAD5 expression. *BioMed Research International*.

[28] Xiao L., Jiang L., Hu Q., Li Y. (2017). MicroRNA-133b ameliorates allergic inflammation and symptom in murine model of allergic rhinitis by targeting Nlrp3. *Cellular Physiology and Biochemistry*.

[29] Powers J. T., Tsanov K. M., Pearson D. S. (2016). Multiple mechanisms disrupt the _let-7_ microRNA family in neuroblastoma. *Nature*.

[30] Shakeri A., Ghanbari M., Tasbandi A., Sahebkar A. (2021). Regulation of microRNA-21 expression by natural products in cancer. *Phytotherapy Research*.

[31] Niu Z., Fu M., Li Y., Ren H., Zhang X., Yao L. (2022). Osthole alleviates pulmonary vascular remodeling by modulating microRNA-22-3p mediated lipid metabolic reprogramming. *Phytomedicine*.

[32] Liu W., Xie G., Yuan G. (2021). 6'-O-Galloylpaeoniflorin attenuates Osteoclasto-genesis and relieves Ovariectomy-induced osteoporosis by inhibiting reactive oxygen species and MAPKs/c-Fos/NFATc1 signaling pathway. *Frontiers in Pharmacology*.

[33] Gao J., Song L., Xia H., Peng L., Wen Z. (2020). 6'-O-galloylpaeoniflorin regulates proliferation and metastasis of non-small cell lung cancer through AMPK/miR-299-5p/ATF2 axis. *Respiratory Research*.

[34] Song L., Peng L., Hua S. (2018). miR-144-5p enhances the radiosensitivity of non-small-cell lung cancer cells via targeting ATF2. *BioMed Research International*.

[35] Song L., Luo J., Wang H. (2022). Legionella pneumophila regulates host cell motility by targeting Phldb2 with a 14-3-3*ζ*-dependent protease effector. *eLife*.

[36] Song L., Li D., Gu Y. (2016). MicroRNA-126 targeting _PIK3R2_ inhibits NSCLC A549 cell proliferation, migration, and invasion by regulation of PTEN/PI3K/AKT pathway. *Clinical Lung Cancer*.

[37] Song L., Li D., Li X. (2017). Exposure to PM2.5 induces aberrant activation of NF-*κ*B in human airway epithelial cells by downregulating miR-331 expression. *Environmental Toxicology and Pharmacology*.

[38] Song L., Xie Y., Li C. (2021). TheLegionellaeffector SdjA is a bifunctional enzyme that distinctly regulates phosphoribosyl ubiquitination. *MBio*.

[39] Song L., Li D., Gu Y., Li X., Peng L. (2016). Let-7a modulates particulate matter (</=2.5 mum)-induced oxidative stress and injury in human airway epithelial cells by targeting arginase 2. *Journal of Applied Toxicology*.

[40] Furuya R., Hu H., Zhang Z., Shigemori H. (2012). Suffruyabiosides a and B, two new monoterpene diglycosides from moutan cortex. *Molecules*.

[41] Yao C. W., Piao M. J., Kim K. C. (2014). Cytoprotective effects of 6'-O-galloylpaeoniflorin against ultraviolet B radiation-induced cell damage in human keratinocytes. *In Vitro Cellular & Developmental Biology. Animal*.

[42] Chai P., Tian J., Zhao D. (2016). GSE1 negative regulation by miR-489-5p promotes breast cancer cell proliferation and invasion. *Biochemical and Biophysical Research Communications*.

[43] Li Y., Ma X., Wang Y., Li G. (2017). miR-489 inhibits proliferation, cell cycle progression and induces apoptosis of glioma cells via targeting SPIN1-mediated PI3K/AKT pathway. *Biomedicine & Pharmacotherapy*.

[44] Lin Y., Liu J., Huang Y., Liu D., Zhang G., Kan H. (2017). microRNA-489 plays an anti-metastatic role in human hepatocellular carcinoma by targeting matrix Metalloproteinase-7. *Translational Oncology*.

[45] Li J., Qu W., Jiang Y. (2016). miR-489 suppresses proliferation and invasion of human bladder cancer cells. *Oncology Research*.

[46] Chen X., Wang Y. W., Xing A. Y. (2016). Suppression of SPIN1-mediated PI3K–Akt pathway by miR-489 increases chemosensitivity in breast cancer. *The Journal of Pathology*.

[47] Wu H., Xiao Z., Zhang H., Wang K., Liu W., Hao Q. (2014). MiR-489 modulates cisplatin resistance in human ovarian cancer cells by targeting Akt3. *Anti-Cancer Drugs*.

[48] Silke J., Vucic D. (2014). IAP family of cell death and signaling regulators. *Methods in Enzymology*.

[49] Werner T. A., Tamkan-Ölcek Y., Dizdar L. (2016). Survivin and XIAP: two valuable biomarkers in medullary thyroid carcinoma. *British Journal of Cancer*.

[50] Lin F., Ghislat G., Luo S., Renna M., Siddiqi F., Rubinsztein D. C. (2015). XIAP and cIAP1 amplifications induce Beclin 1-dependent autophagy through NF*κ*B activation. *Human Molecular Genetics*.

[51] Emery I. F., Gopalan A., Wood S. (2017). Expression and function of ABCG2 and XIAP in glioblastomas. *Journal of Neuro-Oncology*.

[52] Obexer P., Ausserlechner M. J. (2014). X-linked inhibitor of apoptosis protein - a critical death resistance regulator and therapeutic target for personalized cancer therapy. *Frontiers in Oncology*.

[53] Deveraux Q. L., Takahashi R., Salvesen G. S., Reed J. C. (1997). X-linked IAP is a direct inhibitor of cell-death proteases. *Nature*.

[54] Deveraux Q. L., Reed J. C. (1999). IAP family proteins--suppressors of apoptosis. *Genes & Development*.

